# Radiomics Model Based on Enhanced Gradient Level Set Segmentation Algorithm to Predict the Prognosis of Endoscopic Treatment of Sinusitis

**DOI:** 10.1155/2022/9511631

**Published:** 2022-06-22

**Authors:** Yabing Li, Ye Tao

**Affiliations:** ^1^Department of Otolaryngology, Lujiang People's Hospital, Lujiang 231500, China; ^2^School of Life Medicine, University of Science and Technology of China, Hefei, 230026 Anhui, China

## Abstract

**Methods:**

Computed tomography (CT) images of sinusitis in 91 patients were collected. By introducing boundary gradient information into the edge detection function, the sensitivity of the level set model to the boundary of different intensities of lesions was adjusted to obtain accurate segmentation results. After that, the segmented CT image was imported into Mazda texture analysis software for feature extraction. Three dimensionality reduction methods were used to screen the best texture features. Four analysis methods in the B11 module were used to calculate the misclassified rate (MCR).

**Results:**

The segmentation algorithm based on an enhanced gradient level set has good segmentation results for sinusitis lesions. The radiomics results show that the raw data analysis method under the Fisher dimensionality reduction method has a low MCR (25.27%).

**Conclusion:**

The enhanced gradient level set segmentation algorithm can segment sinusitis lesions accurately. The radiomics model effectively predicts the prognosis of endoscopic treatment of sinusitis.

## 1. Introduction

Sinusitis is a common disease in otorhinolaryngology, and the incidence rate is increasing year by year [1–3]. Its clinical manifestations are primarily purulent runny nose, nasal obstruction, and headache, similar to upper respiratory tract infection. Some will also show systemic symptoms such as poor appetite, listlessness, and even fever. In addition, children's resistance is low, immunity is also poor, sinus mucosa and nasal obstruction are pretty fragile, and their ability to apply to the outside world is also very poor. Hence, sinusitis is easy to occur [4]. Correct diagnosis and reasonable treatment can improve the quality of life, reduce the burden of society and family, and reduce the complications caused by sinusitis. Surgery is an essential means of clinical treatment of the disease. Due to the complex structure of the nasal cavity, the operation space of traditional radical surgery is small, and the damage to the nasal structure is extensive. Hence, its curative effect is not ideal. Endoscopic sinus surgery is a minimally invasive surgery assisted by a nasal endoscope [5–7]. This surgery has the characteristics of minor trauma, high polyp resection rate, and fast postoperative recovery [8].

Endoscopic sinus surgery has become the first choice for treating sinusitis with poor drug control. However, the depth of treatment is not easy to grasp, which will affect the treatment. Computed tomography (CT) imaging technology is widely used in nasal cavity and paranasal sinus diseases and has become a meaningful way to diagnose sinusitis. However, some sinusitis is still challenging to identify in clinical practice. This phenomenon has caused some difficulties in judging the disease and surgery. In 2012, Lambin et al. [9] first produced the definition of radiomics, a large number of quantitative information features such as the size, shape, texture, edge, and function of lesions are screened from sectional images. These informations are then transformed into collectible data and analyzed to diagnose the nature of lesions and assist imaging doctors in making the most accurate diagnosis [10–13].

Due to the complex anatomical structure of paranasal sinus and low contrast with surrounding tissues, it is difficult to obtain prior knowledge to help realize paranasal sinus segmentation. This brings great difficulties to the segmentation of the paranasal sinus. As a model-based contour extraction algorithm, the level set method has attracted extensive attention in biomedical image segmentation. The level set has good segmentation characteristics as a geometric active contour model algorithm. Still, it often cannot get satisfactory segmentation results for medical images with high segmentation target complexity and poor contrast with the background [14–16]. Therefore, this study uses the CT radiomics model based on the enhanced gradient level set segmentation algorithm to predict and analyze the prognosis of endoscopic treatment of sinusitis.

## 2. Material and Methods

### 2.1. General Data

A total of 91 patients with chronic sinusitis treated in the Department of Otolaryngology of our hospital from Jun 2019 to Mar 2020 were analyzed retrospectively. There were 64 males and 27 females. The age ranged from 17 to 82 years, with an average of (53.32 ± 13.02) years. This study was reviewed and approved by the hospital medical ethics committee.

Inclusion criteria: (1) Meet the clinical diagnosis of sinusitis. (2) Receive CT scan.. (3) There were apparent symptoms of nasal congestion, runny nose, and decreased olfactory function, and the symptoms were not improved after more than four weeks of conservative treatment. (4) The patients were informed of the study content and signed the consent form. Exclusion criteria: (1) Patients with congenital nasal diseases, atrophic rhinitis, intracranial diseases, and craniocerebral trauma. (2) Acute and chronic respiratory tract infection.

### 2.2. CT Examination

The coronal or horizontal scanning was performed with GE proseed AI single row spiral CT. Coronal scanning: the scanning line is perpendicular to the hard palate, from the anterior wall of the frontal sinus to the posterior wall of the sphenoid sinus, with a layer thickness of 5 mm. Horizontal scanning: taking the line parallel to the orbit and ear as the baseline, the scanning range was from the upper edge of the frontal sinus to the alveolar process of maxilla. Scanning parameters: voltage 120 kv, current 100 mA, scanning speed 1.5, pitch 1 : 1. Matrix 512 × 512. Image window: the width of soft tissue window is 20HU and the window level is 40HU. The width of the bone window is 1500hu and the window level is 40HU.

### 2.3. Endoscopic Sinus Surgery

All patients received endoscopic sinus surgery, and the specific operation plan was determined according to the preoperative examination results. The patient took the supine position, used local anesthesia, observed the structure of the nasal cavity under nasal endoscopy, determined the position of nasal polyps, and performed rhinoplasty and correction of nasal septum deviation according to the specific situation in the nasal cavity after resection of nasal polyps. After that, the sulcus process shall be removed and the maxillary sinus orifice shall be opened. If necessary, the expansion operation can be carried out to altogether remove the polyp tissue and purulent secretion. According to the CT examination results, the frontal sinus orifice and sphenoid sinus orifice shall be opened as appropriate after the operation. After trimming the surgical field of vision, the nasal cavity was rinsed with normal saline, and the surgical cavity was filled with expanded sponge soaked with hormone drugs to stop bleeding. Take out the sponge 1-2 days after the operation and rinse the nasal cavity. Antibiotics were used for 3 days after operation, and regular reexamination and follow-up were carried out.

### 2.4. Level Set Algorithm Based on Enhanced Gradient

For CT images of sinusitis, due to its own particularity, the focus is located in the surrounding tissues, there is a weak boundary, and the changes of the focus boundary gradient of different CT images are complex and diverse. In the edge detection of the CT region of sinusitis, there are usually many irregular lines, which directly interfere with the accuracy of contour curve in the recognition of lesion boundary. The existing level set algorithms usually need complex image information statistics or repeated experiments in practical operation. When using level set algorithm to segment sinusitis lesions, the speed and accuracy of active contour evolution are the focus of attention. Applying the edge detection function *g* in the level set algorithm makes the zero level set close to the direction in which *G* becomes smaller, and the contour curve stays at the edge of the target to be segmented when the value of *G* is the smallest. This requires the level set to accelerate the evolution in a certain range with small gradient and decelerate the evolution and convergence in the range of high gradient. In this study, the edge detection function is defined as follows to adjust its sensitivity to edges with different intensities.

(1) $$\begin{array}{c} g=e^{-{\left|\nabla G_{\sigma }*I\right|}^{2}+1/\left|I_{0}^{2}/{\left|\nabla G_{\sigma }*I\right|}^{2}-1\right|+1}. \end{array}$$

*I*_0_ is the preset gradient value of lesion boundary. When the image gradient |∇*I*| approaches the lesion boundary gradient *I*_0_, |∇*G*_*σ*_∗*I*|^2^ + 1/|*I*_0_^2^/|∇*G*_*σ*_∗*I*|^2^ − 1| + 1 tends to the maximum and *g* decreases to the minimum, so that the level set evolution curve can selectively and quickly approach the lesion contour.

Figure 1 shows the edge detection function curve of enhanced gradient level set segmentation algorithm. It can be seen from the figure that the edge detection function constructed in this study has faster descent and convergence speed, and targeted control of the curve descent inflection point. The evolution of the level set *ε*, which controls the evolution of the zero level set to the main driving energy of the target edge to be segmented, drives the contour curve to move to the target boundary under the influence of the edge detection function g:

(2) $$\begin{array}{c} \varepsilon_{g,\lambda ,\mu }\left(\Phi \right)=\lambda \int g\delta \left(\Phi \right)\left|\nabla \Phi \right|dxdy+v\int gH\left(-\Phi \right)dxdy. \end{array}$$

The first term on the right is the length energy term, and the second term is the area energy term, where *λ* and *v* are constants and *λ* > 0, *δ* is a univariate Dirac function, and H is the Heaviside function. Equation (2) fully considers the tumor boundary information and improves the sensitivity of level set evolution to boundary gradient. *I*_0_ value is close to the gradient value of lesion boundary, which can effectively improve the accuracy and evolution speed of level set segmentation for specific targets.

### 2.5. Evaluation of Lesion Segmentation Results

The performance of the segmentation algorithm can be evaluated by some quantitative indexes. When evaluating the level set segmentation algorithm combined with clinical needs, this study focuses on whether the focus area of sinusitis can be segmented accurately and quickly. Taking the manual segmentation results of radiologists as the gold standard, this paper uses two evaluation indexes of tpvf and fpvf to count the semi-automatic segmentation results of lesion area.

(3) $$\begin{array}{c} \text{TPVF}=\frac{\left|C_{o}^{b}\cap C_{t}^{b}\right|}{\left|C_{t}^{b}\right|}\times 100\%,\\ \text{FPVF}=\frac{\left|C_{o}^{b}\cap C_{t}^{b}\right|}{\left|C_{\text{d}}-C_{t}^{b}\right|}\times 100\%, \end{array}$$

where *C*_*o*_^*b*^ and *C*_*t*_^*b*^ are the level set segmentation results and the doctor's manual segmentation gold standard, respectively, and *C*_*d*_ is the region for analysis. In this paper, the region of interest of the original CT image is taken. TPVF indicates the percentage of correctly segmented tissue. FPVF is the evaluation index of over segmentation or false segmentation.

### 2.6. Imaging Treatment of Sinusitis Lesions

Firstly, the horizontal axial plain and enhanced images of the largest level of the target lymph node of each patient (the plain and enhanced images must be the same level) were selected and imported into the open source Mazda 4.6 software (http://www.eletel.p.lodz.pl/Mazda/) in DICOM format from the PACS system. After the image is imported, the gray level standardization processing is carried out first to reduce the influence of different brightness and contrast of the image on the gray value. Then, the region of interest (ROI) was drawn in the target lymph node by manual segmentation method. The edge of ROI was 1-2 mm away from the edge of the lesion to avoid calcification, peripheral blood vessels, and other areas. After the lesion was outlined, a total of 275 texture features including run length matrix, gray co-occurrence matrix, gray histogram, absolute gradient, wavelet transform, and autoregressive model were extracted by Mazda software.

After that, through Mazda's three screening methods, namely, Fisher coefficient (Fisher), classification error probability, combined with average correlation coefficient (POE+ACC) and mutual information (MI), 10 best texture features are screened out by each method, and a total of 30 best texture features are screened out. Then, B11 module is used for feature analysis. B11 module includes four analysis methods: original data analysis, principal component analysis, linear classification analysis, and nonlinear classification analysis. The final analysis results are expressed by the misclassified rate (MCR). The lower the MCR, the better the classification benefit of the model.

### 2.7. Statistical Analysis

The results were statistically analyzed by SPSS 20. Chi square test was performed on the general data, and K-S test was used to determine the normality of the data. All data were in accordance with normal distribution, and the differences between groups were analyzed by single factor *t*-test. The difference was statistically significant (*P* <0.05).

## 3. Result

### 3.1. Segmentation Results

Firstly, a rectangular region containing head and neck tumors in the patient's CT image was manually selected during the experiment. Then, any closed curve (such as a triangle) in the lesion in the ROI is selected as the initial contour of level set evolution (Figure 2).

When using the enhanced gradient level set algorithm to process CT images, the gradient value at the lesion boundary is significantly higher than that at other locations of the lesion. This paper first sets a target window at the lesion using this feature. The gray gradient value in the window can be roughly divided into two parts: the smaller gradient inside the lesion and soft tissue and the more significant gradient at the boundary. Therefore, the average value *x* and mean square deviation *y* of the gray gradient in the window can be calculated. Then, take *x* + *y* as the threshold and bring the average value of gray gradient higher than the threshold as the lesion boundary gradient I. The figure shows the segmentation results. The active contour did not converge in the lesion or leak at the weak boundary and achieved good segmentation results.

### 3.2. Radiomics Processing

Mazda is used to extract the features of CT images, and a total of 256 texture features were extracted. Then, Fisher, POE + ACC, and MI are used to reduce the dimension of texture features, and 10 best features are selected, respectively, as shown in Figure 3.

Figure 4 shows the analysis results of RDA, PCA, LDA, and NDA under the Fisher dimensionality reduction method. Among them, 1 represents good prognosis, 2 represents poor prognosis. The greater the separation of 1 and 2, the better the identification effect of this analytical method. From Table 1, the raw data analysis method under the Fisher dimensionality reduction method has a low MCR (25.27%).

## 4. Discussion

There will be mucosal congestion, edema, and enlarged turbinate when there is nasal inflammation. This phenomenon can easily cause the runny nose to flow to the pharynx and drip behind the nose, stimulate the pharynx, and have symptoms such as adherence, retching, nausea, and bad breath [17, 18]. These symptoms usually lead to missed diagnosis and misdiagnosis, delaying the best time for treatment. With the development of modern medicine, endoscopic technology is more and more widely used in the clinic [19]. Endoscopic sinus surgery for patients with chronic sinusitis can reduce surgical trauma and speed up postoperative recovery.

Imaging methods provide a noninvasive diagnostic idea. Compared with ordinary X-ray film, the CT of paranasal sinus has obvious advantages [20, 21]. X-ray film has only reference value for the diagnosis of sinusitis in children. Relevant reports show that the misdiagnosis rate reaches 80%, because the skull is thin and lacks obvious contrast with soft tissue in density, so it is easy to be misdiagnosed [22]. CT scan can overcome the deficiency of X-ray film and can display tissues with different densities, such as mucosa, bone, and pus. At the same time, CT scanning can reduce the number of additional rays received by children and reduce the loss of robotic ball tubes.

The CT-based radiomics method extracts texture features only based on CT value data, which is relatively fast, simple, and easy to use [16, 23]. At present, there have been some studies on the prognosis prediction of diseases based on radiomics [24, 25]. There are various algorithms in disease diagnosis and prognosis [26, 27]. Heo et al. [28] found that the machine learning algorithm based on clinical information (NIHSS score, past medical history, laboratory examination, etc.) can improve the prediction of long-term prognosis of patients with ischemic stroke. Xie et al. [29] conducted gradient boosting machine learning to predict the prognosis based on the imaging, epidemiological, and clinical data of 512 patients with acute stroke. The results showed that the accuracy of predicting the adverse prognosis was 87.7%.

The level calculation method based on the enhanced gradient proposed in this paper uses the edge detection function assuming the preset boundary gradient value, adjusts the sensitivity of the level set model to the lesion boundary, and effectively improves the influence of local gradient texture on the evolution of level set. Mazda's results show that RDA analysis under the Fisher dimensionality reduction method has good efficiency, and its misjudgment rate is only 25.27%.

## 5. Conclusions

To sum up, the enhanced gradient level set algorithm has a good segmentation effect for sinusitis lesions. The NDA analysis under the MI dimensionality reduction method has a low misjudgment rate in the follow-up texture analysis. The results indicate that the texture parameters under the MI screening have a good predictive effect on the prognosis of endoscopic sinus treatment, and can help patients with effective treatment.

## Figures and Tables

**Figure 1:** Edge detection function curve of enhanced gradient level set segmentation algorithm.

**Figure 2:** Segmentation results of augmented gradient-based level set method in CT image. (a) Initial contour. (b) Evolution contour (blue line) and the gold standard (red line). (c) Segmented lesion area.

**Figure 3:** Best texture parameters under three dimensionality reduction methods. (a) Fisher. (b) POE+ACC. (c) MI.

**Figure 4:** Analysis results under the Fisher dimensionality reduction method. (a) RDA. (b) PCA. (c) LDA. (d) NDA.

**Table 1:** Misclassified rate result.

	RDA	PCA	LDA	NDA
Fisher	23/91 (25.27%)	24/91 (26.37%)	40/91 (43.96%)	26/91 (28.57%)
POE+ACC	35/91 (38.46%)	32/91 (35.16%)	37/91 (40.66%)	26/91 (28.57%)
MI	35/91 (38.46%)	39/91 (42.86%)	36/91 (39.56%)	26/91 (28.57%)

## Data Availability

The data used to support the findings of this study are available from the corresponding author upon request.
